# Observation on the Effect of Rehabilitative Physical Training on Ice and Snow Sports Injury under Ultrasound Examination

This article has been retracted.

**DOI:** 10.1155/2022/2931686

**Published:** 2022-08-08

**Authors:** Yang Wang, Yongzhi Zhou

**Affiliations:** Physical Culture Institute, Jilin Normal University, Siping, Jilin 136000, China

## Abstract

In order to solve the problem of rehabilitative physical training on ice and snow sports injuries, the author proposed an observation method using ultrasonography to be proposed. This method selects patients with anterior talofibular ligament injury treated in a hospital, forty-nine patients who did not undergo conventional rehabilitation under the surveillance of sports medicine ultrasound were set as the control group, a total of 49 patients with anterior talofibular ligament injury who underwent rehabilitation treatment under the monitoring of sports medicine ultrasound were selected as the experimental group, and the clinical efficacy of the two groups of patients was retrospectively analyzed, in order to discuss the application value of sports medicine ultrasound in the rehabilitation of anterior talofibular ligament injury. The results showed that comparing the rehabilitation effect, ankle function score, and daily living ability of the two groups of patients, the experimental group was better than the control group. Comparing the thickness of ligament and effusion between the two groups, the experimental group was also better than the control group, and the difference was statistically significant (*P* < 0.05). Ultrasound medical examination can help doctors to effectively judge the degree of injury and recovery of patients, and doctors can adjust the treatment plan in time according to the examination results and formulate an effective rehabilitation plan, which can greatly shorten the recovery time of patients, improve the treatment effect, promote the functional recovery of the ankle joint, and reduce the occurrence of complications.

## 1. Introduction

Competitive sports are often accompanied by sports injuries, which are one of the biggest obstacles for athletes to create good results and have a negative impact on athletes' normal training, competitive competition, and life psychology and even affect their sports career [1]. Years of training, coupled with the strict technical and movement requirements of ice and snow events, have resulted in common injuries to the lower back, knees, ankles, and other parts of the athletes; this type of injury has the characteristics of inconspicuous pathogenesis, lack of targeted treatment, poor efficacy, and difficult to cure, which seriously affects the career and physical and mental health of athletes in winter sports [2]. Chinese scholars have done a lot of research on winter sports injuries, but there are few data on the application of personalized rehabilitation therapy for sports injuries, and it is mainly based on conventional treatment after the injury occurs and lacks specificity [3]. How to minimize the pain and injury of athletes, create better competitive performance, and specific treatment plan, this is a topic that many scholars at home and abroad pay great attention to.

The vast majority of sports injuries are soft tissue injuries, and the corresponding diagnostic methods rely on clinical examinations, such as palpation, percussion, and functional tests, which depend to a certain extent on the experience of clinicians, ultrasound examination can provide a direct and objective diagnostic basis of sonographic images [4]. The application of ultrasound to the musculoskeletal system has been tried by scholars in various historical periods, but it was really applied in the field of orthopedics, especially the diagnosis of muscle, ligament, and soft tissue injuries after the 1980s. In the past five years, there have been more and more researches on this aspect, covering all countries in the world. In my country, there have also been reports on the application of ultrasound to bone and soft tissue injuries, but no systematic report on the use of ultrasound in sports injuries has been found, the author introduces the diagnosis and treatment of nearly 49 cases of sports injuries by using ultrasonography, and through clinical and related diagnostic techniques, according to the experimental data, the effect of rehabilitative physical training on ice and snow sports injury under ultrasound examination was observed [5].

## 2. Literature Review

Winter sports have higher technical requirements for athletes, and athletes are likely to overload their sports parts during day-to-day single-event training, resulting in lumbar muscle strain, ankle injury, knee joint injury, etc. [6]. In winter sports athletes, muscle strains and ligament strains occur during exercise, and the patients have the highest probability of injury to the lower back, knees, and ankles, followed by shoulders, wrists, and legs [7]. During daily training or competition of athletes, the body is often kept at a low temperature, and the muscles are easily stiffened rapidly, when doing strenuous exercise to contract the muscles, the muscles are strained due to excessive force, and the auxiliary tissues around the muscles may also be damaged [8]. Because of the less blood vessels and muscles in the knee and ankle joints, easy fatigue, and slow recovery, athletes are prone to sports injuries in these two parts [9]. Bullen et al. found that the injury rate of athletes was 55.2% in daily training and 36.8% in event competition [10]. In addition, different sports and different injuries of athletes are also related. Majumder and Deen believed that sports injuries of athletes in ice sports mainly occurred in the lower back and limb joints [11]. Therefore, in the process of exercising, athletes have greater psychological pressure, and the speed and impact force are more intense than general exercise [12]. Further analysis found that joint sprains accounted for the highest proportion of major injuries in athletes, followed by muscle strains [13]. Winter sports have the highest rate of sprains, followed by abrasions, falls, and bruises. Winter sports characteristics are related to the type of injury that occurs. Ice athletes have high technical requirements, high speed, and great difficulty and are prone to falls and collisions, resulting in falls or bruises [14]. Snow athletes are prone to bumps or falls when they encounter road obstacles during training or competition. In addition, due to the low temperature in winter, if athletes in winter sports do not keep warm or other reasons, the blood flow in the body is not smooth, and frostbite on the face, hands, and feet is prone to occur [15].

Taking patients who visited the orthopedics department of a hospital from January 2020 to January 2021 as an example, there was no statistical difference in the general population data between the two groups (*P* > 0.05) (Table 1).

By comparing the main sports injury parts of the two groups of patients, it was found that the lower back, knee, and ankle joints had the highest incidence of injury, followed by the shoulder, wrist, and leg, and the chest and abdomen had the lowest injury probability. There was no significant difference in the main sports injury sites between the two groups (*P* > 0.05) (Table 2).

The statistics and comparison results of the main injury types of the two groups of patients are shown in Table 3. Among the injury types, joint sprains accounted for the highest proportion, followed by muscle strains, ligament strains and myofasciitis injuries were also more common, with the lowest rates of abrasions and frostbite. There was no significant difference in the main types of sports injuries between the two groups (*P* > 0.05).

Ultrasound technology has shown many advantages in the diagnosis and treatment of athletes' rehabilitation physical training (Figure 1), mainly because it is noninvasive, economical, and real-time, it is popular with athletes and coaches, because this technology can solve problems quickly without affecting training [16], no preparation is required before the examination, and the examination results are immediately available; during the examination, the coaches can directly participate in the understanding of the situation, and there is no need to rest after the examination, therefore, it is meaningful to add ultrasound equipment as a sports injury research department and a front-line training base.

## 3. Methods

### 3.1. General Information

Select the anterior talofibular ligament injury treated in a hospital from January to December 2020, forty-nine patients who did not undergo conventional rehabilitation under the surveillance of sports medicine ultrasound were set as the control group, and a total of 49 patients with anterior talofibular ligament injury who underwent rehabilitation treatment under the surveillance of sports medicine ultrasound from January to December 2020 were selected as the experimental group for retrospective analysis [17]. Among them, there were 31 males and 18 females in the experimental group, with an average age of (30.97 ± 5.16) years. Among them, there were 32 patients with right ligament injury, 21 males and 11 females, and 17 left ligament injuries, 10 males and 7 females. In the control group, there were 30 males and 19 females with an average age of (31.01 ± 5.39) years. Among them, there were 34 patients with right ligament injury, 22 males and 12 females, and 15 left ligament injuries, and 8 male cases and 7 females. The comparison of general data showed that the difference was not statistically significant (*P* > 0.05), which was comparable.

### 3.2. Inclusion and Exclusion Criteria

1. Inclusion criteria

(1) Approved by the ethics committee of the hospital. (2) All patients and their families signed the informed consent. (3) All patients underwent stress imaging X-ray films before treatment, and the posterior opening of the ankle joint was ≥6 mm, which was in line with the clinical criteria for anterior talofibular ligament injury. The fracture site of the patients is often associated with other medical conditions.

(2) Exclusion criteria

(1) Patients are with mental illness. (2) Patients are with disorders of consciousness and communication. (3) Patients are with coagulation disorders. (4) Patients are with major diseases of other organs. (5) Patients are with contraindications to related drugs and treatment. (6) Fracture location patients are with other severe diseases [18]

### 3.3. Experimental Method

1. Control group

The patients were treated with conventional rehabilitation therapy: (1) ankle mobilization was performed for the patient, 30 min/time, 1 time/d; continuous treatment for 30 times was a course of treatment; according to the specific conditions of the patients, 2 to 3 courses of treatment were performed, and the manipulation was grade 3 to 4. (2) If the patient undergoes surgical treatment, the patient should be elevated after surgery, and an ice pack should be used to cool the ankle joint, 2 times a day, for 3 to 5 days, and 1 day after the operation, the patient should be helped to perform ankle pump exercise through the protection of the ankle joint brace, and the exercise content includes straight leg raises and stepping on a bottle of wine on the affected foot. 2 days after the operation, the patients were instructed to perform ankle dorsiflexion, rotation, and active plantar flexion, 10 min/time, 3-7 times/d, so that the patient could reach the maximum range of motion of the ankle within 2 weeks. On the 7th day after operation, incomplete weight-bearing training with crutches was used to gradually increase the intensity of foot resistance exercises, followed by weight-bearing walking training; after 3 weeks of operation, the patient could walk without crutches; 3 months after surgery, you can basically return to normal exercise capacity [19]. Passive exercise can be added if necessary, but the intensity of exercise should be well controlled, and the exercise should be done gradually to avoid re-injury. If there is fluid accumulation in the ankle joint of the patient, the exercise intensity of the patient should be appropriately reduced, and timely treatment should be performed; if necessary, puncture and fluid extraction can be performed. (3) Perform computer intermediate frequency therapy, 2 times/d, mainly for the function of the patient's tibialis anterior muscle and gastrocnemius muscle. In addition, high-power short-wave and pulsed magnetic therapy and electric weight loss gait therapy and air pressure therapy are used, 1-2 times/d. Continue treatment for 1 month.

(2) Test group

The patients were supplemented with sports medicine ultrasound examination on the basis of the control group: (1) the high-frequency ultrasound diagnosis grading of ligament injury was analyzed by ultrasonography, 25 cases (51.02%) of grade I injury (contusion) occurred, the ligament was thickened, with good continuity, and the echo was reduced and uneven. In 17 cases (34.69%) of grade II injury (partial laceration), part of the ligament was interrupted and thinned, the echo was reduced, and there was a fissure-like or sheet-like hypoechoic area, with or without effusion in the joint cavity. In 7 cases (14.29%) of grade III injury (complete laceration), the continuity of the ligament was completely interrupted, the broken end was separated, the echo was reduced, the surrounding echo was disordered, and dynamic scanning showed that the ligament tension disappeared [20]. (2) The doctor adjusts the patient's rehabilitation training intensity and methods according to the examination results, formulates a targeted rehabilitation training plan, and conducts the rehabilitation training before and after the patient's treatment. Ultrasonography was performed at 1 month, 2 months, and 3 months, respectively, to observe the swelling, exudation, and repair of the patient's ligament and adjust the treatment plan according to the results.

### 3.4. Observation Indicators

(1) Comparing the rehabilitation effects of the two groups of patients after 6 months of treatment, the echoes of the fully recovered ligaments were uniform, and the structure was flat and smooth. The pain and swelling of the ankle joint disappeared completely, the patient walked normally, and the range of motion of the joint was normal. Ultrasound examination of incompletely recovered ligaments showed bilateral contrast thickening, incomplete structure, abnormal joint mobility, and pain when walking. (2) The thickness of the anterior talofibular ligament and the thickness of the effusion were compared between the two groups of patients before and after treatment. (3) The ankle function scores of the two groups of patients after 3 months of treatment were compared, the Biard-Jackson scale was used to evaluate the ankle joint function, the excellent ankle function was 96-100 points, the good was 91-95 points, the average was 81-90 points, and the poor was 81 points or less. (4) The daily living ability of the two groups before and 3 months after treatment was compared, and the activity of daily living scale (ADL) was used to evaluate the daily living ability, the full score was 100 points, the higher the score, the better the living ability, the stronger.

### 3.5. Statistical Processing

The article uses SPSS 22.0 statistical software to process and analyze, the count data is expressed by (*n*, %), the *χ*^2^ test is carried out, the measurement data is described by ($\bar{x}\pm s$), and the *t* test is used. *P* < 0.05 indicates that the difference is statistically significant.

#### 3.5.1. *t*-Test

*t*-test is a hypothesis test method established by British statistician W.S. Gosset in 1908 based on the principle of *t*-distribution, and it is often used to compare the means of two small samples in measurement data. Theoretically, the application condition of the *t* test is that the samples are from a normally distributed population, and the variance of the two populations is equal when the means of the two samples are compared. But in actual work, it deviates slightly from the above conditions, as long as its distribution is unimodal and approximately normal distribution, it can also be applied.

There are three types of commonly used *t*-tests: (1) single-sample *t*-test: it is used to infer whether the overall mean represented by the sample mean and the known overall mean are statistically significant. When the number of samples is small (*n* < 60) and the overall standard deviation is unknown, the *t*-test is used; conversely, when the number of samples is large or the number of samples is small and the overall standard deviation is known, the *u* test can be used. (2) Paired specimen *t*-test: it is suitable for the comparison of the means of the two specimens in the paired design, and attention should be paid to whether the two specimens are paired design data when selecting [21]. The commonly used paired design data mainly have the following three situations: two homogeneous subjects receive two different treatments. The same subject or two parts of the same specimen received different treatments, respectively. The results of the same subject before and after treatment were compared. (3) Two independent samples *t*-test: also known as grouped *t*-test, it is suitable for the comparison of the means of two samples in a completely random design. Unlike the paired *t*-test, before performing the two-independent *t*-test, the homogeneity of variance test must also be performed on the two groups of data. If the sample is small and the variance is homogeneous, the *t*-test is used; otherwise, if the variance is unequal, the corrected *t*-test (*t*-test) is used or use data transformation methods (such as logarithm, square root, and reciprocal) to make the two groups of data have homogeneity of variance and then carry out *t*-test or use nonparametric test. In addition, when the number of samples in the two groups is large (*n*1, *n*2 > 50), the calculation of the *t*-test is cumbersome, and the *u* test can be used.

## 4. Results and Discussion

### 4.1. Comparison of Rehabilitation Effects between the Two Groups of Patients

The rehabilitation effect of the patients in the experimental group was better than that of the patients in the control group, and the difference was statistically significant (*P* < 0.05), as shown in Table 4.

### 4.2. Comparison of the Thickness of the Anterior Talofibular Ligament and the Thickness of the Effusion between the Two Groups of Patients before and after Treatment

The values of the experimental group were better than those of the control group, and the difference was statistically significant (*P* < 0.05), see Table 5.

### 4.3. Comparison of Ankle Function Scores between the Two Groups of Patients

The ankle joint score of the experimental group was higher than that of the control group, and the difference was statistically significant (*P* < 0.05), as shown in Table 6.

### 4.4. Comparison of Daily Living Ability between the Two Groups of Patients

The living ability of the patients in the experimental group was better than that in the control group, and the difference was statistically significant (*P* < 0.05), as shown in Figure 2.

### 4.5. Discussion

With the continuous development of ultrasound technology, it has been at a high level, especially the sports medicine ultrasound technology has made great progress, its application in the examination and evaluation of soft tissue injuries has higher value, and doctors can obtain more objective data and indicators through this examination to improve their evaluation level [22]. When a patient has ligament injury, sports medicine ultrasonography can be used to determine the degree of tear of the patient's anterior talofibular ligament, and the treatment plan can be formulated according to the examination results. This examination method is used as an auxiliary means during the treatment and rehabilitation of patients, which can monitor the rehabilitation status of patients, which is of great significance for the timely adjustment of rehabilitation methods. Doctors can provide effective rehabilitation guidance in the process of patient recovery, shorten the patient's recovery time, and speed up the patient's recovery. The author compared the rehabilitation effect, ankle function score, and daily living ability of the two groups of patients; and the experimental group was better than the control group. Comparing the thickness of ligament and effusion between the two groups, the experimental group was also better than the control group, and the difference was statistically significant (*P* < 0.05). In summary, in the treatment of patients with anterior talofibular ligament injury, the use of sports ultrasound medical examination can help doctors to effectively judge the degree of injury and recovery of patients, and doctors can adjust the treatment plan in time according to the examination results and formulate an effective rehabilitation plan, which can greatly shorten the patient's rehabilitation time, improve the treatment effect, promote the functional recovery of the ankle joint, and reduce the occurrence of complications.

## 5. Conclusion

The author proposes to use ultrasound examination to observe the effects of rehabilitative physical training on ice and snow sports injuries, by dividing the patients into experimental group and control group for experimental data analysis, and it is concluded that the experimental group is superior to the control group. With the continuous development of ultrasound technology, it has been at a high level, especially the sports medicine ultrasound technology has made great progress, its application in the examination and evaluation of soft tissue injuries has higher value, and doctors can obtain more objective data and indicators through this examination and improve their evaluation level. Therefore, it can be determined that this method can effectively improve the treatment effect of patients, reduce pain, relieve psychological pressure, and be applied to the rehabilitation of winter sports system injuries.

## Figures and Tables

**Figure 1:** Rehabilitation physical training.

**Figure 2:** Comparison of daily living ability between the two groups of patients (score, $\bar{x}\pm s$).

**Table 1:** Comparison of general data of the two groups of patients.

Project	Personalization group (*n* = 40)	Regular group (*n* = 40)	*t*/*x*^2^	*P* value
Gender: male female	14/26	12/28	1.747	0.533
Age	17.7 ± 2.1	17.2 ± 1.9	0.825	0.876
Average training time/year	4.3 ± 2.0	4.8 ± 2.5	1.443	0.452

**Table 2:** Comparison of main injury sites in the two groups of patients.

Injury site	Personalization group (*n* = 40)		Regular group (*n* = 40)		*P* value
	Number of cases/cases	Rate/%	Number of cases/cases	Rate/%	
Lower back	11	27.5	12	30.0	0.468
Knee and hip joints	13	32.5	15	37.5	0.332
Shoulder and wrist joints	6	15.0	4	10.0	0.317
Head and face	2	5.0	1	2.5	0.462
Chest and abdomen	1	2.5	0	0.0	−
Legs	5	12.5	4	10.0	0.428
Other	2	5.0	4	10.0	0.347

**Table 3:** Comparison of main injury types between the two groups of patients.

Damage type	Personalization group (*n* = 40)		Regular group (*n* = 40)		*P* value
	Number of cases/cases	Rate/%	Number of cases/cases	Rate/%	
Joint sprain	12	30.0	12	30.0	1.000
Muscle strain	8	20.0	10	25.0	0.419
Myofasciitis	4	10.0	3	7.5	0.283
Joint contusion	3	7.5	4	10.0	0.507
Belt strain	7	17.5	7	17.5	0.462
Bruises	2	5.0	1	2.5	0.404
Bruise	3	7.5	2	5.0	0.393
Frozen	1	2.5	1	2.5	1.000

**Table 4:** Comparison of rehabilitation effects between the two groups of patients (cases (%)).

Group	Recover completely	General recovery	Not fully recovered
Test group (*n* = 49)	46 (93.88)	10 (51.23)	3 (6.12)
Control group (*n* = 49)	39 (79.59)	9 (12.34)	10 (20.41)
*χ* ^2^ value	4.3460		
*P* value	0.0371		

**Table 5:** Comparison of the thickness of the anterior talofibular ligament and the thickness of the effusion between the two groups of patients before and after treatment (mm, $\bar{x}\pm s$).

Group	Ligament thickness		Effusion thickness	
	Before therapy	After treatment	Before therapy	After treatment
Test group (*n* = 49)	4.37 ± 0.59	3.67 ± 0.57	7.54 ± 2.17	2.82 ± 0.67
Control group (*n* = 49)	4.61 ± 0.63	4.03 ± 0.65	7.49 ± 2.13	5.20 ± 1.78
*t* value	1.8444	2.7622	0.1091	8.3006
*P* value	0.0686	0.0070	0.9134	0.0000

**Table 6:** Comparison of ankle function scores between two groups of patients (points, $\bar{x}\pm s$).

Group	Biard-Jackson score	
	Before therapy	After treatment
Test group (*n* = 49)	62.35 ± 6.71	89.71 ± 2.17
Control group (*n* = 49)	62.76 ± 6.05	80.45 ± 1.98
*t* value	0.3010	20.9098
*P* value	0.7641	0.0000

## Data Availability

The data used to support the findings of this study are available from the corresponding author upon request.
